# Prediction of Prognostic Risk Factors in Patients with Invasive Candidiasis and Cancer: A Single-Centre Retrospective Study

**DOI:** 10.1155/2022/7896218

**Published:** 2022-06-02

**Authors:** Jingyi Li, Yaling Li, Yali Gao, Xueli Niu, Mingsui Tang, Chang Fu, Zihan Wang, Jiayi Liu, Bing Song, Hongduo Chen, Xinghua Gao, Xiuhao Guan

**Affiliations:** ^1^Department of Dermatology, The First Hospital of China Medical University, 110001 Shenyang, China; ^2^Center for Translational Medicine Research and Development, Shen Zhen Institutes of Advanced Technology, Chinese Academy of Science, Shenzhen, Guangdong 518055, China; ^3^Department of Dermatology, The First Affiliated Hospital, Sun Yat-sen University, Guangzhou 510080, Guangdong, China

## Abstract

**Background:**

Invasive candidiasis is a common cancer-related complication with a high fatality rate. If patients with a high risk of dying in the hospital are identified early and accurately, physicians can make better clinical judgments. However, epidemiological analyses and mortality prediction models of cancer patients with invasive candidiasis remain limited.

**Method:**

A set of 40 potential risk factors was acquired in a sample of 258 patients with both invasive candidiasis and cancer. To begin, risk factors for *Candida albicans* vs. non-*Candida albicans* infections and persistent vs. nonpersistent *Candida* infections were analysed using classic statistical methods. Then, we applied three machine learning models (random forest, logistic regression, and support vector machine) to identify prognostic indicators related to mortality. Prediction performance of different models was assessed by precision, recall, *F*1 score, accuracy, and AUC.

**Results:**

Of the 258 patients both with invasive candidiasis and cancer included in the analysis. The median age of patients was 62 years, and 95 (36.82%) patients were older than 65 years, of which 178 (66.28%) were male. And 186 (72.1%) patients underwent surgery 2 weeks before data collection, 100 (39.1%) patients stayed in ICU during hospitalisation, 99 (38.4%) patients had bacterial blood infection, 85 (32.9%) patients had persistent invasive candidiasis, and 41 (15.9%) patients died within 30 days. The usage of drainage catheter and prolonged length of hospitalisation are the dominant risk factors for non-*Candida* albicans infections and persistent *Candida* infections, respectively. Risk factors, such as septic shock, history of surgery within the past 2 weeks, usage of drainage tubes, length of stay in ICU, total parenteral nutrition, serum creatinine level, fungal antigen, stay in ICU during hospitalisation, and total bilirubin level, were significant predictors of death. The RF model outperformed the LR and SVM models. Precision, recall, *F*1 score, accuracy, and AUC for RF were 64.29%, 75.63%, 69.23%, 89.61%, and 91.28%.

**Conclusions:**

In this study, the machine learning-based models accurately predicted the prognosis of cancer and invasive candidiasis patients. The algorithm could be used to help clinicians in high-risk patients' early intervention.

## 1. Background

Invasive candidiasis, defined as bloodstream and deep-seated infections of the genus Candida, is prone to occur in patients with prolonged hospitalisation, HPV (human papillomavirus) infection, immunotherapy, and organ transplantation [1, 2]. Despite the development of treatments for Candidaemia over the last decade, it remains extremely lethal, with an attributable mortality rate ranging from 5% to 70% [3]. A recent 12-year epidemiological study of Candidaemia in the Paris region showed that people admitted to the ICU and those with haematological malignancies or solid tumours had a significantly increased risk of death, ranging from 29.4% to 51.3% [4]. And outside the ICU, overall death at day 30 was significantly higher in patients with solid tumours (34.9%) than in those with haematological caners (29.4%) or no malignancy (22.5%).

Delayed antifungal treatment is considered the main cause of poor prognosis in candidemia, leading to a 3-fold increase in mortality [5]. Part of the reason for this comes from the low sensitivity of fungal cultures of blood, urinary tissue, and other body fluids (38-50%) [6, 7]. Therefore, risk factor analysis and predictive modelling are critical for preventing such diseases or identifying patients who should be treated early.

Compared with traditional statistical methods, machine learning (ML) focuses on improving prediction accuracy, whereas the former is concerned with the correlations between variables [8]. Based on supervised machine learning algorithms, computers can process tens of thousands of instances, replete with feature-to-label mapping, to develop a model that generalises the data, and process a never-before-seen input [9]. Furthermore, ML takes into account the complete spectrum of available data, whereas traditional statistical methods tend to prioritise factors [10]. In diverse medical domains such as disease diagnosis, prognosis prediction, drug development, and customised therapy, machine learning is now frequently applied [11–13].

In this study, we collected the data of 258 patients with cancer with invasive candidiasis, described their clinical characteristics and biochemical tests in detail, and eventually used different machine learning models to identify prognostic factors related to death.

## 2. Methods

### 2.1. Data Collection

In this study, the data of 258 patients with both cancer and invasive candidiasis were collected from the electronic database of the First Hospital of China Medical University from January 2013 to January 2018. Patient's age, sex, medical history (basic disease and medication history), length of hospital stay, laboratory tests, and some other clinical features were included. It is important to emphasize that patient cultured fungal cultures were obtained from blood, pleural fluid, ascites fluid, and peritoneal dialysis fluid. Each hospitalisation was a separate incident for the same patient. The particular criteria for selection, definition, and abbreviation can be found in the previous literature [14].

### 2.2. Model Development

#### 2.2.1. Phase 1: Machine Learning Dataset Preprocessing

To reduce the impact of meaningless values, we firstly fill the mean and zero for numerical and categorical missing data, respectively. Then, all remaining data were modified by using “one-hot encoding (OHE)” [15].

#### 2.2.2. Phase 2: Outlier Detection

Due to the small size of the dataset, each sample has a crucial impact in the training process of the model. We choose Density-based Spatial Clustering of Applications with Noise (DBSCAN) technique to identify outliers and limit the influence of erroneous samples on the model, which is a common outlier identification approach based on clustering [16]. DBSCAN's fundamental idea is to identify dense regions, which may be estimated based on the number of items around a particular point, and to remove outliers, which are points that do not belong to any cluster. In DBSCAN, clusters are determined by two parameters: epsilon (*ε*) and minimum points (minPts), which defined each cluster must satisfy that the number of samples within the *ε* radius is at least minPts. This means that when *ε* is larger or minPts is smaller, the final number of outlier is less; while when *ε* is smaller or minPts is larger, the number of outlier is more. In this experiment, the final parameters are determined by the grid method. Considering the small size of the data in this experiment, the number of outlier needs to be controlled within a certain range, and we use the logistic regression model as the baseline model with 5-fold cross-validation for evaluating the quality of the data set after eliminating the outliers.

#### 2.2.3. Phase 3: Data Segmentation

The dataset was randomly divided into training and test sets (7 : 3 ratio). The training set is to train prediction model, whereas the test set is to evaluate the trained model. Such data segmentation was repeated 5 times to test the performance of each predictive model.

#### 2.2.4. Phase 4: Oversampling

Because our dataset had a large difference between positive (died, 40) and negative (alive, 214) sample numbers, there was a need to balance the dataset. By creating artificial data, “oversampling” is an effective method that can be used to reduce variations within imbalanced data, such as Synthetic Minority Oversampling Technique (SMOTE) [17]. It can create artificial data based on neighbouring data from datasets with small sample size, thus increasing the number of the datasets. By using SMOTE, we expand the training set data from 177 to 298 subjects, with 149 positive subjects. Finally, the prediction model was trained using these 298 subjects.

#### 2.2.5. Phase 5: Model Development and Evaluation

To better predict patient outcomes, we tested and evaluated three machine learning algorithms (RF, LR, and SVM) [18]. Precision, recall, specificity, *F*1 score, and accuracy were the evaluation metrics. The flow chart for model development is shown in Figure 1.

### 2.3. Statistical Analysis

The IBM SPSS Statistics for iOS version 26.0 software (IBM Corp., Armonk, NY, USA) was used for statistical analysis. Median and quartile ranges (*M*(*P*25, *P*75)) were used to describe the quantitative data. When the data was normally distributed, it was analysed using the *t*-test for comparisons. When the data was nonnormally distributed, it was analysed using the Mann–Whitney test. And the chi-square test was use for the comparisons of qualitative data.

## 3. Results

### 3.1. Clinical Features of Patients

A total of 258 patients with both cancer and invasive candidiasis were included in this study, including patients with solid tumours (243/258, 94.9%) and haematologic malignancies (15/258, 5.81%). Most patients with solid tumours had digestive system malignancies, such as gastric cancer (66/258, 25.6%), colon cancer (46/258, 17.8%), rectal cancer (34/258, 13.2%), pancreatic cancer (22/258, 8.5%), small intestine cancer (19/258, 7.4%), cholangiocarcinoma (15/258, 5.8%), liver cancer (8/258, 3.1%), and oesophageal cancer (6/258, 2.3%) (Figure 2). More detailed information can be found in Supplementary Table 1. The median age of the patients in this study was 62 years, with 95 (36.82%) of them being above 65. There were also more male patients (171/258, or 66.28%) than female patients (87/258, or 33.7%). In addition, 186 (72.1%) patients underwent surgery 2 weeks before data collection, 100 (39.1%) patients stayed in ICU during hospitalisation, 99 (38.4%) patients had bacterial blood infection, 85 (32.9%) patients had persistent invasive candidiasis, and 41 (15.9%) patients died within 30 days. These characteristics indicated that the patients were immunocompromised. During hospitalisation, 100 (39.1%) patients were administered three or more types of antibiotics, 32 (12.4%) patients were administered immunosuppressants, and 4 (1.5%) patients were administered glucocorticoids. The majority of patients had surgery, with 225 (87.2%), 158 (61.7%), and 160 (62.0%) patients using urinary catheters, stomach tubes, and central venous lines, respectively. More detailed information can be found in Supplementary Table 2.

In this study, we also found that the probability of *C. parapsilosis* infections was the highest (104/258, 40.3%), followed by *C. guilliermondi* (83/258, 32.2%), *C. albicans* (33/258, 12.8%), *C. tropicalis* (18/258, 7.9%), *C. glabrata* (17/258, 6.6%), and *C. krusei* (3/258, 1.2%) infections (Figure 3).  Figure 4 depicts the spread of blood bacterial infection in 99 patients. A total of 37 species of bacteria were isolated. *Acinetobacter baumannii* (40/231, 17.3%) was the most common pathogenic bacteria, followed by *Escherichia coli* (27/231, 11.7%), *Enterococcus faecium* (23/231, 10.0%), *Staphylococcus aureus* (18/231, 7.8%), *Pseudomonas aeruginosa* (17/231, 7.4%), and *Klebsiella pneumoniae* (16/231, 6.9%). Supplementary Table 3 contains more detailed information.

### 3.2. Antifungal Susceptibility Testing

Supplementary Table 4 entails the antifungal susceptibility results of *Candida* spp. isolated from 249 patients with cancer with invasive candidiasis. It is noteworthy that resistance to *amphotericin B* was not observed in all 249 isolates. *C. parapsilosis*, *C. guilliermondii*, and *C. glabrata* all showed susceptibility to antifungal agents, while their sensitivity varied. *C. tropicalis* exhibited the strongest antifungal resistance, especially to fluconazole (3/17, 17.6%), voriconazole (3/17, 17.6%), and itraconazole (2/17, 11.8%). In contrast, *C. glabrata* isolates were highly susceptible to fluconazole (7/16, 43.8%), itraconazole (6/16, 37.5%), and voriconazole (5/16, 31.3%) in a dose-dependent manner. Overall, itraconazole (20/249, 8.0%) showed the highest dosage dependence and the resistance rate of fluconazole was the highest (6/249, 2.4%).

### 3.3. Risk Factors for *Candida albicans* and Non-*Candida albicans* Infections

The comparison of demographics and clinical characteristics of patients with *C. albicans* and non-*Candida albicans* infections is summarized in Table 1. First, the presence of gastric tube (42.4% versus 60%, *P* = 0.018), drainage tube (57.58% versus 84%, *P* < 0.001), and total parenteral nutrition (75.8% versus 92.9%, *P* = 0.002) was more frequent in patients with non-*Candida albicans* infections. In addition, compared with patients with *C. albicans* infections, patients with non-*Candida albicans* infections also stayed in the hospital for a longer duration (30 versus 39 days, respectively, *P* = 0.024). In terms of laboratory inspections, the leukocyte, neutrophil, and lymphocyte counts were higher in patients with non-*Candida albicans* infections, with the median of leukocyte and neutrophil counts exceeding the normal value.

### 3.4. Analysis of Risk Factors in Patients with Persistent and Nonpersistent *Candida* Infections

Table 2 summarized the difference in demographics and clinical characteristics between patients with persistent and nonpersistent Candida. Invasive mechanical ventilation and prolonged hospital or ICU stays raised the risk of recurrent Candida infection in patients. The leukocyte, neutrophil, and lymphocyte counts were higher in patients with persistent Candida infection. However, patients who underwent surgery in the past 2 weeks were unlikely to have persistent Candida infection, which may be related to the use of antibiotics before and after surgery.

### 3.5. Prediction of Risk Factors for Death via Machine Learning

As mentioned before, we firstly collected all useful information of 258 samples (Supplementary Table 5). After data processing, we used DBSCAN ( *ε* = 180 and minPts = 30) to delete outliers (three alive samples and one died sample). Remaining samples were randomly divided into training set (177 samples) and test set (77). Because of the large gap in the number of alive (149 samples) and died (28 samples) cases within the training set, we used SMOTE to expand the number of death samples. Consequently, in the training set, we obtained a total of 298 samples in the training set (alive : died = 149 : 149). Then, we applied three different ML models (RF, LR, and SVM) to predict the mortality of patients. All steps above were randomly replicated five times. The final performance evaluation is the average of 5 results, which are expressed in Table 3 and Figure 5. RF with the highest value of precision (0.69), recall (0.75), *F*1 score (0.72), accuracy (0.89), and AUC (0.91) showed the best performance when compared with other prediction models. Therefore, RF was selected to rank the importance of each risk factor. As shown in Table 4, the most predictive characteristics of death in patients with cancer accompany with invasive candidiasis were septic shock, history of surgery within the past 2 weeks, usage of drainage tubes, length of stay in ICU, total parenteral nutrition, serum creatinine level, fungal antigen, stay in ICU during hospitalisation, and total bilirubin level.

## 4. Discussion

Invasive candidiasis is a common and devastating complication among cancer patients. The clinical features, pathogen distribution, and risk factors of mortality of 258 cancer patients with invasive candidiasis were investigated in this study. We discovered that 72.1% patients had surgery within the past 2 weeks, and 39.1% were admitted to the ICU, indicating a higher frequency of IFD in the surgical ICU, which is consistent with the findings of other study [19]. Invasive candidiasis shows significant geographical and demographic heterogeneity [20]. Several studies on invasive fungal infections in the Asia-Pacific region have reported that *C. albicans* infections continue to be the most common (36–41.3%) [21, 22]. Conversely, in the United States of America, the infection rate of *C. albicans* infection is dropping, and *C. glabrata* infection is increasing, accounting for one-third or more of candidiasis cases [23]. According to our statistical findings, *C. parapsilosis* infections were the most prevalent, followed by *C. guilliermondi*, *C. albicans*, *C. tropicalis*, *C. glabrata*, and *C. krusei* infections.

In our study, amphotericin B was the most sensitive antifungal agent. Because *Candida* spp. isolated from 249 patients were not resistant to it based on antifungal susceptibility testing. This result is consistent with that of another study on antifungal susceptibility of *Candida* spp. [24]. *C. tropicalis* was of particular interest because it was the most resistant to fluconazole (3/17, 17.6%), voriconazole (3/17, 17.6%), and itraconazole (2/17, 11.8%). This finding is line with the results of another study on azole resistance in *C. tropicalis* from China, which showed that 12.8% (65/507) of the strains were resistant to fluconazole [25]. And it was speculated that the resistance was mainly related to the ERG11 mutation in *C. tropicalis*. However, a study from Iran showed that no accountable mutations in the ERG11 gene could be detected in 64 *C. tropicalis* blood isolates [26].

Previous studies have demonstrated that total parenteral nutrition is an independent risk factor of NAC bloodstream infections [27, 28]. Similarly, a higher incidence of NAC infection was found in this study in patients with gastric tubes, drainage tubes, total parenteral nutrition, and longer stay in hospital. Furthermore, a study by Gong et al. showed that drainage tube usage was an independent risk factor in *C. albicans* infection [29]. They also found no significant difference in the length of stay in the hospital between patients with *C. albicans* and NAC infections. In terms of biochemical parameters, our results revealed that the levels of white blood cells, neutrophils, and lymphocytes were lower in patients with NAC infections than in patients with *C. albicans* infection. This finding is consistent with that of a study by Chi et al., which suggested that neutropenia was predictive of NAC infections. But, to date, the association of neutropenia with invasive fungal disease remains unclear [30]. Because the heterogeneity of the study population often leads to different results [8, 30, 31]. In this study, prolonged hospital stays, admission to the ICU, and the use of invasive mechanical ventilation increased the likelihood of persistent candidiasis infections, which is consistent with the findings of previous studies [32].

In recent years, machine learning techniques have gotten a lot of interest in the pharmaceutical industry. To develop and test a predictive model for Candidaemia in cancer patients, Liu et al. used machine learning algorithms to analyse clinical data from 186,404 cancer patients. All machine learning models (AUROC 0.771-0.889) outperformed statistical models (AUROC 0.677), with RF being the best (AUROC 0.889) [33]. In this study, the overall mortality rate was 15.89%, which is lower than that reported in other studies [34–36], i.e., between 31.9% and 58%. Consequently, depending on the characteristics of our dataset, our prediction models specifically combined ML with DBSCAN-based outlier detection and oversampling technique SMOTE. These are the key novelty of our study. Without DBSCAN and SMOTE, the precision, recall, *F*1 score, accuracy, and AUC for RF were 0.86, 0.4, 0.55, 0.97, and 0.69. Liu et al. used machine learning algorithms to analyse clinical information from 186,404 cancer patients to develop and validate a predictive model for Candidaemia in cancer patients. Their results showed that all machine learning models outperformed the statistical models, with RF performing the best.

Of all predictors, septic shock was the most significant factor. This finding is consistent with that of previous studies, which showed that invasive candidiasis complicated by septic shock is almost fatal [11, 32, 34, 37]. Failure to initiate appropriate antifungal therapy and manage the source of infection in a timely manner was the main cause of shock [38]. Patients who do not receive antifungal therapy within 30 days of identifying Candida infection are more likely to die than those who receive effective antifungal therapy [39]. In this study, the predictors also included a history of surgery within the past 2 weeks, drainage tube use, length of ICU stay, total parenteral nutrition, serum creatinine levels, fungal antigens, ICU stay during hospitalisation, and total bilirubin levels. Although it is now widely recognised that prompt antifungal therapy is critical, deciding the best time to initiate antifungal therapy remains challenging. A study on the efficacy and safety of prophylactic fluconazole in surgical patients revealed that invasive candidiasis occurred in 2 of 23 patients treated with fluconazole and 7 of 20 patients treated with placebo in high-risk surgical patients [40]. A report on ESCMID guidelines also recommended the use of fluconazole for the prevention of invasive candidiasis in patients who had recently undergone abdominal surgery and had recurrent gastrointestinal perforations or anastomotic fistulas [41]. Furthermore, an elevated serum creatinine level represents diminished renal function and can increase mortality in patients, although they may develop renal failure.

The retroactive aspect of our study limited its findings. The time of the beginning and end of interventions was not documented in the medical records of the patients, and the inclusion of biochemical indicators varied among the medical records. Further examination of the risk and prognostic factors for invasive candidiasis in patients with different tumour types was not performed because the study was a single-centre study, and the number of patients with haematological tumours included was smaller than the number of patients with solid tumours.

## 5. Conclusion

We report for the first time epidemiological data on patients with both cancer and invasive candidiasis. Based on the DBSCN and SMOTE algorithms, we use the RF model with high accuracy predict the mortality risk factors. The main predictors of death are septic shock, history of surgery within the past 2 weeks, usage of drainage tubes, length of stay in ICU, total parenteral nutrition, serum creatinine level, fungal antigen, stay in ICU during hospitalisation, and total bilirubin level.

## Figures and Tables

**Figure 1:** Flow chart of machine learning.

**Figure 2:** Tumour types of 258 patients.

**Figure 3:** Candida species in 258 patients.

**Figure 4:** The distribution of blood bacterial infection in 99 patients.

**Figure 5:** Receiver operating characteristic curve of different machine learning models.

**Table 1:** Risk factors for Candida albicans and non-Candida albicans infections.

	Candida albicans % (*n* = 33)	Non-Candida albicans % (*n* = 225)	Statistic	*P* value
Male	23 (69.70%)	148 (65.78)	0.445	0.657
Age (years)^a^	61.00 (56.00, 69.00)	63.00 (54.00, 70.00)	-0.191	0.848
Length of stay (days)^a^	30.00 (23.00, 46.00)	39.00 (28.00, 62.00)	2.253	0.024
Length of stay in ICU^a^	0.00 (0.00, 4.00)	1.00 (0.00, 8.00)	1.658	0.097
Solid tumour	33 (100%)	213 (94.67%)	1.359	0.174
Diabetes	7 (21.21%)	25 (11.11%)	1.644	0.100
Pancreatitis^b^	1 (3.03%)	1 (0.44%)	—	0.240
Total parenteral nutrition	25 (75.76%)	209 (92.89%)	3.164	0.002
Renal failure	1 (3.03%)	11 (4.89%)	—	1
Recent surgery (within 2 weeks)	20 (60.61%)	166 (73.78%)	1.575	0.115
Use immunosuppressants^b^	6 (18.18%)	26 (11.56%)	—	0.267
ICU	17 (51.52%)	83 (36.89%)	1.611	0.107
Hypoproteinemi^a^	27 (81.82%)	161 (71.56%)	1.238	0.216
Invasive mechanical ventilation	14 (42.42%)	70 (31.11%)	1.295	0.195
Urinary catheter	31 (93.94%)	194 (86.22%)	1.240	0.215
Gastric tube	14 (42.42%)	144 (64.00%)	2.376	0.018
Central venous catheter	20 (60.61%)	140 (62.22%)	0.179	0.858
Drainage catheter	19 (57.58%)	189 (84.00%)	3.586	<0.001
Endotoxic shock^b^	5 (15.15%)	22 (9.78%)	—	0.360
Multiple hospitalisations within 2 years (>2 times)	22 (66.67%)	140 (62.22%)	0.493	0.622
Persistent fungal infection	12 (36.36%)	73 (32.44%)	0.447	0.655
Serum albumin level^a^ (g/l)	27.80 (24.60, 30.80)	25.90 (22.60, 29.00)	-1.659	0.097
Serum creatinine level^a^ (*μ*mol/L)	57.00 (45.00, 72.00)	67.00 (40.00, 88.00)	0.990	0.322
Leukocyte count^a^ (10^9/l)	6.54 (4.56, 9.52)	12.26 (7.46, 14.19)	4.829	<0.001
Total bilirubin level^a^ (*μ*mol/l)	14.00 (8.80, 26.70)	17.30 (10.60, 56.10)	0.999	0.318
Neutrophil count^a^ (10^9/l)	5.30 (3.73, 7.95)	9.22 (5.13, 11.68)	3.591	<0.001
Lymphocyte count^a^ (10^9/l)	0.64 (0.44, 0.90)	0.85 (0.53, 1.13)	2.017	0.044
CRP^a^ (mg/l)	85.70 (58.55, 124.25)	95.40 (76.10, 182.00)	1.322	0.186
PCT^a^ (ng/ml)	0.46 (0.24, 1.09)	0.96 (0.24, 3.46)	1.174	0.240
CD4	305.00 (150.00, 463.5)	234.00 (159.00, 317.00)	0.570	0.569
CD8	152.00 (98.00, 227.50)	110.00 (74.00, 289.00)	0.297	0.767
CD3	472.00 (252.50, 700.50)	398.00 (241.00, 634.00)	0.388	0.698
CD4/CD8	1.37 (0.91, 2.49)	1.93 (1.08, 3.13)	-0.661	0.509

Note: ^a^ is described by median and quartile, and the statistic was the *Z* value; other items were described as numbers (*n* − %), and the statistic was the *χ*^2^ value, ^b^ statistic was the Fisher *χ*^2^ value.

**Table 2:** Risk factors in patients with persistent and nonpersistent Candida infections.

	Persistent Candida infection (%) (*n* = 85)	Nonpersistent Candida infection (%) (*n* = 74)	Statistic	*P* value
Male	59 (69.41%)	44 (59.46%)	1.310	0.190
Age (years)^a^	63.00 (56.00, 70.00)	61.00 (54.00, 66.75)	1.575	0.115
Length of stay (days)^a^	39.00 (30.00, 62.00)	32.00 (25.00, 44.75)	3.048	0.002
Length of stay in ICU^a^	3.00 (0.00, 12.00)	0.00 (0.00, 3.00)	2.761	0.006
Diabetes	16 (18.82%)	8 (10.81%)	—	0.187
Total parenteral nutrition	78 (91.76%)	68 (91.89%)	0.029	0.977
Renal failure	7 (8.24%)	3 (4.05%)	—	0.340
Recent surgery (within 2 weeks)	52 (61.18%)	56 (75.68%)	2.102	0.036
Use immunosuppressants within the past 30 days^b^	13 (15.29%)	11 (14.86%)	—	1
Stay in ICU during hospitalisation	46 (54.12%)	27 (36.49%)	2.225	0.026
Hypoproteinemi^a^	67 (78.82%)	51 (68.92%)	1.424	0.154
Invasive mechanical ventilation	41 (48.24%)	23 (31.08%)	2.200	0.028
Urinary catheter	74 (87.06%)	62 (83.78%)	0.586	0.558
Gastric tube	54 (63.53%)	44 (59.46%)	0.526	0.599
Central venous catheter	60 (70.59%)	45 (60.81%)	1.299	0.194
Drainage catheter	70 (82.35%)	61 (82.43%)	0.013	0.990
Septic shock	15 (17.65%)	5 (6.76%)	—	0.054
Multiple hospitalisations within 2 years (>2 times)	58 (68.24%)	51 (68.92%)	0.093	0.926
Serum albumin level^a^ (g/l)	27.40 (24.50, 29.30)	28.40 (25.10, 31.63)	-1.500	0.133
Serum creatinine level^a^ (*μ*mol/L)	58.00 (42.00, 82.00)	57.50 (47.25, 68.75)	-0.040	0.968
Leukocyte count^a^ (10^9/l)	7.86 (5.35, 11.12)	5.77 (4.13, 9.02)	3.234	0.001
Total bilirubin level^a^ (*μ*mol/l)	15.50 (11.00, 33.30)	14.20 (7.40, 24.73)	1.877	0.061
Neutrophil count^a^ (10^9/l)	6.34 (4.00, 9.11)	4.61 (3.07, 7.39)	2.624	0.009
Lymphocyte count^a^ (10^9/l)	0.79 (0.59, 1.06)	0.56 (0.39, 0.75)	3.605	<0.001
CRP^a^ (mg/ml)	96.55 (66.88, 122.75)	84.90 (61.60, 121.50)	0.574	0.566
PCT^a^ (ng/ml)	0.53 (0.26, 1.10)	0.45 (0.24, 1.45)	0.459	0.646

Note: ^a^ is described by median and quartile, and the statistic was the *Z* value; other items were described as numbers (*n* − %), and the statistic was the *χ*^2^ value. ^b^ statistic was the Fisher *χ*^2^ value.

**Table 3:** Performance evaluation for the prediction models.

Model	Precision	Recall	*F*1 score	Accuracy	AUC
Random Forest	0.69	0.75	0.72	0.89	0.91
Logistic regression	0.43	0.83	0.57	0.81	0.86
Support vector machine	0.24	0.83	0.38	0.57	0.67

**Table 4:** Feature importance rank.

Feature	Index
Endotoxic shock	0.101668
Recent surgery (within 2 weeks)	0.067329
Total parenteral nutrition	0.058851
Drainage catheter	0.056403
Length of stay in ICU^a^	0.050194
Stay in ICU during hospitalisation	0.045371
Fungal antigen	0.042123
Serum creatinine level	0.037023
Leukocyte count	0.030745
Total bilirubin level	0.028947

## Data Availability

The data supporting the findings of this study from the corresponding author upon request. If someone wants to request the data from this study, please contact Xiuhao Guan.

## Supplementary Materials

Supplementary 1 Supplementary Table 1: tumour types of 258 patients.

Supplementary 2 Supplementary Table 2: detailed clinical data of 258 patients.

Supplementary 3 Supplementary Table 3: types of bacterial infection in 258 patients.

Supplementary 4 Supplementary Table 4: antifungal susceptibility results of 258 patients.

Supplementary 5 SU Supplementary Table 5: raw data of 258 patients.
